The article "Inhibition of miR-15a-5p Promotes the Chemoresistance to Pirarubicin in Hepatocellular Carcinoma via Targeting eIF4E" was retracted in 2023. Reasons: signs of a paper mill; suspected computer-generated content; unreliable results or conclusions; concerns about the data.

# Inhibition of miR-15a-5p Promotes the Chemoresistance to Pirarubicin in Hepatocellular Carcinoma via Targeting eIF4E

**DOI:** 10.1155/2021/6468405

**Published:** 2021-11-13

**Authors:** Ying Zhang, Qingsong Tie, Zhiwei Bao, Zhi Shao, Lan Zhang

**Affiliations:** Jianhu County People's Hospital, Yancheng, 224700 Jiangsu, China

## Abstract

Chemoresistance has become a primary hurdle in the therapeutic outcome of hepatocellular carcinoma. Substantial evidences have demonstrated that microRNAs (miRNAs) are closely associated with the chemoresistance of hepatocellular carcinoma (HCC). Our investigation is aimed at testifying the influence of microRNA-15a-5p (miR-15a-5p)/eukaryotic translation initiation factor 4E (eIF4E) on hepatocellular carcinoma resistance to pirarubicin (THP). In our study, miR-15a-5p expression was increased in THP-treated HepG2 cells. Downregulation of miR-15a-5p blocked cell growth and elevated cell apoptosis of HepG2 cells treated with THP. Moreover, eIF4E was verified as a direct target of miR-15a-5p by binding its 3′-UTR, which was confirmed by luciferase report experiment. Additionally, eIF4E was negatively associated with the miR-15a-5p expression in HepG2 cells. Mechanically, eIF4E was proven as a specific downstream of miR-15a-5p and mediated the effects of miR-15a-5p on cell viability and apoptosis of HepG2 cells treated with THP. These findings supported that miR-15a-5p facilitated THP resistance of hepatocellular carcinoma cells by modulating eIF4E, thus providing an experimental basis that miR-15a-5p might act as a novel diagnostic target in hepatocellular carcinoma resistance to THP.

## 1. Introduction

Hepatocellular carcinoma (HCC) has been regarded as one of the most common malignant tumors in the world with about 600,000 deaths annually [1]. In addition, because of local invasion and intrahepatic metastasis, the recurrence rate of hepatocellular carcinoma patients is very high [2]. Even if radical treatment is used, the prognosis of patients with advanced hepatocellular carcinoma is often poor due to tumor diffusion and invasion, and the 5-year survival rate is less than 5% [3]. At present, the treatment methods for hepatocellular carcinoma include surgery, radiotherapy, chemotherapy, and targeted molecular therapy. However, on the one hand, these treatment methods cannot completely remove the smallest residual cancer cells, including small lesions and tumor metastasis; on the other hand, drug resistance and adverse effects usually exist during treatment [4, 5]. Moreover, cisplatin, carboplatin, cyclophosphamide, 5-fluorouracil, vincristine, and other drugs commonly used in chemotherapy can cause one or more side effects, such as alopecia, nephrotoxicity, myelosuppression, anorexia, and reproductive toxicity [6–8]. Therefore, it is particularly urgent to find a new treatment for hepatocellular carcinoma.

Drug resistance is a critical issue in improving outcome of chemotherapy in live cancer. Two medications in the first line, sorafenib, a multikinase inhibitor and lenvatinib, a multitarget tyrosine kinase vascular endothelial growth factor receptor (VEGFR) and fibroblast growth factor receptor (FGFR) inhibitor, are currently used for the treatment of advanced live cancer. Previous study demonstrated that hedgehog (Hh) signalling components were detected in 50%-70% of specimens in advanced live cancer, indicating that Hh signalling activation in live cancer is common. Studies have implicated Hh signalling plays an important role in enhancing hepatic carcinogenesis, epithelial-mesenchymal transition (EMT), and invasion. Another study implied that Hh signalling mediates drug resistance through targeting TAP1 in hepatocellular carcinoma [4–8].

To date, doxorubicin (DOX) is still the mostly applied chemotherapeutic in the treatment of intermediate or advanced stage of hepatocellular carcinoma. However, drug-induced chemoresistance in hepatocellular carcinoma is frequently developed during chemotherapy and is a huge hurdle in the cancer treatment [9]. Pirarubicin (THP) is a new generation of anthracycline antitumor drugs, which is a derivative of doxorubicin, and is widely used as a first-line drug in the treatment of hematological malignancies [9]. In recent years, studies have shown that THP has a wide antitumor spectrum and can also be used in the treatment of breast cancer, bladder cancer, ovarian cancer, and other solid tumors [10–12]. At the same time, animal experiments have shown that THP has little effect on the reproductive system [9]. For example, THP could inhibit the growth accompanied by G0/G1 phase cell cycle arrest and cell antiproliferation in hepatocellular carcinoma cells [13]. Therefore, the application of THP in the treatment of hepatocellular carcinoma has a good prospect. However, clinical trials showed that most hepatocellular carcinoma patients were not sensitive to THP, and the specific mechanism was not clear, which greatly limited the clinical application of THP [14]. Thus, exploring the possible mechanisms of the insensitivity of hepatocellular carcinoma patients to THP and finding a new strategy for enhancing the therapeutic effect of THP will provide a new idea for the clinical treatment of hepatocellular carcinoma.

Nowadays, microRNAs (miRNAs), a kind of largely functional transcripts with about 200 nucleotides in length, have been deeply implicated in the development of cancers through functioning as oncogenes or cancer suppressor genes [15, 16]. Notably, some miRNAs have been verified to contribute to the formation of chemoresistance in cancers including hepatocellular carcinoma. For instance, miR-590-5p was high-expressed in 5-Fu-resistant hepatocellular carcinoma patients and hepatocellular carcinoma cells, and knockdown of miR-590-5p improved chemosensitivity to 5-Fu in hepatocellular carcinoma via negatively targeting YAP1 [17]. Downregulation of miR-101 reduced chemosensitivity of HepG2 cells to cisplatin through regulation of DNA-dependent protein kinase catalytic subunit/protein kinase B/mammalian target of rapamycin (DNA-PKcs/Akt/mTOR) pathway [18]. miR-15a-5p is located in the 13q14 region of human chromosome and abnormally expressed in a variety of tumors, such as pancreatic cancer, chronic lymphocytic leukemia, and pituitary tumor [19–22]. Recent report has proven that miR-15a-5p could contribute to apoptosis, autophagy, and cisplatin resistance of non-small-cell lung cancer (NSCLC) via targeting Bcl-2 [23]. In addition, inhibition of miR-15a could restore the Taxol-induced resistance to colon cancer mediated with lncRNA00473 [24]. Nevertheless, the precise functions and corresponding mechanisms of miR-15a-5p in the regulation of THP resistance in hepatocellular carcinoma remain largely unknown. Herein, our intention was to elucidate the biological impacts and associated mechanisms of miR-15a-5p on THP resistance of hepatocellular carcinoma.

## 2. Materials and Methods

### 2.1. Cell Culture and Treatment

HepG2 is a human hepatoma that is most commonly used in drug metabolism and hepatotoxicity studies. HepG2 cells are nontumorigenic cells with high proliferation rates and an epithelial-like morphology that perform many differentiated hepatic functions. HepG2 cells were obtained from Chinese Academy of Science and seeded in RPMI-1640 medium under standard conditions. For cell transfection, miR-15a-5p mimics/inhibitors or pc-eIF4E and the corresponding negative control (NC) vectors were obtained from GenScript (China). HepG2 cells (3 × 10^5^) were maintained in 6-well plates and transfected using Lipofectamine 2000 (Invitrogen). Transfection efficiency was examined by qRT-PCR after 48 h.

### 2.2. CCK-8 Assay

For cell viability assessment, transfected cells were maintained for predetermined times (0 h, 24 h, 48 h, and 72 h), respectively. After treatment, cell viability was examined by CCK-8 kit (Beyotime Biotechnology) based on the protocols. The optical density was detected at 490 nm by microplate reader.

### 2.3. EdU Assay

Transfected cells (2 × 10^3^) were plated for 48 h, incubated with EdU (50 *μ*M) for another 2 h, and fixed with 4% formaldehyde for 30 min. Then, the nuclei were counterstained with DAPI. The EdU-positive cells were monitored under a fluorescence microscope (Olympus) at the magnification of 200x.

### 2.4. Flow Cytometry

Apoptotic cells were evaluated by Annexin V-FITC kit (Beyotime Biotechnology). After 48 h, transfected cells were harvested with trypsin and resuspended in 500 *μ*L binding buffer. Next, samples were treated with Annexin V-FITC (5 *μ*L) and PI (10 *μ*L) in the dark for 15 min. Eventually, cell apoptosis was measured by flow cytometer (BD Biosciences, USA).

### 2.5. qRT-PCR

Total RNA was separated from hepatocellular carcinoma cells by Trizol Reagent (Invitrogen). cDNA was synthesized by TaqMan Reverse Transcription Kit (Applied Biosystems). Routine qRT-PCR was implemented using ABI 7300-fast RT PCR system (Applied Biosystems) with SYBR Green PCR Kit (Qiagen) based on the specifications. Relative expressions of miRNA and mRNA were evaluated by the 2^−*ΔΔC*t^ method with U6 or *β*-actin as internal reference. The primer sequences used were listed as follows: miR-15a-5p forward, 5′-ATCCAGTGCGTGTCGTG-3′ and reverse, 5′-TGCTTAGCAGCACATAAT G-3′; eIF4E forward, 5′-AGGAGGTTGCTAACCCAGAA-3′ and reverse, 5′-CAACAGTATCAAAC TTGGAGATCA-3′; SLC9A1 forward, 5′-TGCCCGGTTTTACTCTCATT-3′ and reverse, 5′-AGGCA AGAAGCTCACCAGTC-3′; KCNT2 forward, 5′-GGCCGTGATGCTGACTGCCG-3′ and reverse, 5′-TCCAGAAGAGAGTCCCCGTGGC-3′; SERINC2 forward, 5′-TAATACGACTCACTATAG-3′ and reverse, 5′-ACATCCACTTTGCCTTTCTC-3′; TATDN3 forward, 5′-CATATGAGCGATAAAATT ATTCAC-3′ and reverse, 5′-GGATCCCTTGTCATCGTCATCACCA-3′; PANK1 forward, 5′-CTAGC AAAATAGGCTGTCCC-3′ and reverse, 5′-GACGATAGTCATGCCCCGCG-3′; *β*-actin forward, 5′-G TCACCTTCACCGTTCCAGTTTT-3 and reverse, 5′-CTTAGTTGCGTTACACCCTTTCTT-3′; and U6 forward, 5′-CTCGCTTCGGCAGCACATA-3′ and reverse, 5′-AACGCTTCACGAATTTGCGT-3′.

### 2.6. Western Blot

Protein was isolated by RIPA lysis buffer and quantified by BCA kit (Beyotime Biotechnology). Protein was extracted by 12% SDS-PAGE and then shifted into PVDF membranes (Millipore, MA, USA). Next, the membranes were interfered with 5% nonfat milk and treated with the primary antibodies overnight at 4°C. Membranes were washed and probed with HRP-conjugated secondary antibody (1 : 2,000, ab6728) for 1 h at room temperature. At last, protein blots were observed by enhanced chemiluminescence kit (ECL, Millipore, Bedford, MA, USA) and quantified using the Image J software (NIH, version 4.3). The primary antibodies were as follows: anti-caspase-3 (1 : 500, ab197202), anti-eIF4E (1 : 500, ab33766), anti-SLC9A1 (1 : 500, ab216573), anti-KCNT2 (1 : 500, ab123543), anti-SERINC2 (1 : 500, ab134312), anti-TATDN3 (1 : 500, ab126654), anti-PANK1 (1 : 500, ab96173), and anti-*β*-actin (1 : 1,000, ab179467). All antibodies were obtained from Abcam (MA, USA).

### 2.7. Target Gene Prediction and Luciferase Reporter Assay

The candidate target gene of miR-15a-5p was predicted with ENCORI and miRwalk, and eIF4E was chosen as a target gene through qPCR and western blot assays. The sequence of wild-type eIF4E (eIF4E-WT) and eIF4E (eIF4E-Mut) was inserted into pmirGLO reporter vector (GenScript, China). Then, pmirGLO-eIF4E-WT/Mut were cotreated with miR-15a-5p mimics or NC into HepG2/THP cells using Lipofectamine 2000 (Invitrogen). The activity of luciferase was examined by luciferase reporter assay system (Promega) and exhibited as firefly luciferase intensity calibrated to Renilla luciferase activity.

### 2.8. Statistical Analysis

Data analysis was implemented by GraphPad Prism 5.0 and presented as mean ± standard deviation (SD). One-way ANOVA followed by Tukey's post hoc analysis was employed to analyze the differences between groups. *P* < 0.05 was indicated to be significant.

## 3. Results

### 3.1. miR-15a-5p Is Upregulated in THP-Treated HepG2 Cells

In order to explore the possible role and underlying mechanisms of miR-15a-5p in chemoresistance of hepatocellular carcinoma, firstly, qRT-PCR was employed to screen the expression profile of miR-15a-5p in HepG2 cells treated with THP. As presented in Figure 1, miR-15a-5p was highly expressed in THP-treated HepG2 cells. These findings depicted that miR-15a-5p was closely implicated in THP chemoresistance of hepatocellular carcinoma.

### 3.2. Downregulation of miR-15a-5p Blocks Cell Growth and Elevates Cell Apoptosis in THP-Treated HepG2 Cells

To figure out the influence of miR-15a-5p in THP chemoresistance of HepG2 cells, HepG2 was transfected with miR-15a-5p inhibitor, and the data of Figure 2(a) illustrated that miR-15a-5p level was sharply diminished in miR-15a-5p inhibitor-transfected cells, revealing the successful depletion of miR-15a-5p. Following the inhibition of miR-15a-5p in HepG2 cells, CCK-8 results hinted a time-dependent reduction in cell viability of HepG2 cells treated with THP (Figure 2(b)). Consistently, EdU assay declared that miR-15a-5p inhibition repressed the proliferative ability of HepG2 cells treated with THP, as reflected by the declined numbers of EdU-positive cells (Figure 2(b)). Besides, the detection of cell apoptosis disclosed that downregulation of miR-15a-5p observably exaggerated the percentage of apoptotic cells of HepG2 cells treated with THP (Figure 2(c)). Furthermore, it was confirmed that miR-15a-5p depletion promoted the expression of apoptosis-related protein including caspase-3 in HepG2 cells treated with THP (Figure 2(d)). Collectively, these outcomes elucidated that interference of miR-15a-5p expression blocked cell growth and elevated cell apoptosis in HepG2 cells treated with THP.

### 3.3. eIF4E Is a Target Gene of miR-15a-5p and Negatively Associated with miR-15a-5p Expression

To ascertain the possible mechanisms of miR-15a-5p, bioinformatics tools including ENCORI and miRwalk were jointly utilized, and a total of 381 intersecting target genes were selected, including eIF4E, SLC9A1, KNCT2, SERINC2, TATDN3, and PANK1, related to chemoresistance. In addition, no obvious difference was existed at mRNA and protein expression levels between NC inhibitor and miR-15a-5p inhibitor groups, except for eIF4E (Figure 3(a)). Moreover, luciferase reporter analysis was employed to validate the interactions between miR-15a-5p and eIF4E. As expected, exogenous expression of miR-15a-5p could distinctly weaken the luciferase activity of 3′-UTR of eIF4E, whereas the inhibitory effect was blocked by mutation on the putative binding sites existed on the 3′-UTR of eIF4E (Figures 3(b) and 3(c)). Furthermore, qRT-PCR and western blot assays were employed to validate eIF4E expression levels in HepG2 cells transfected with miR-15a-5p inhibitor, and the data of Figures 3(d) and 3(e) revealed that the mRNA and protein levels of eIF4E were remarkably upregulated in HepG2 cells transfected with miR-15a-5p inhibitor. Generally, these data suggested that eIF4E may be a potential target gene of miR-15a-5p in hepatocellular carcinoma.

### 3.4. eIF4E Mediates the Effects of miR-15a-5p on the THP Chemoresistance of HepG2 Cells

Having corroborated the negative relation between miR-15a-5p and eIF4E expression in HepG2 cells, the regulatory relationship of miR-15a-5p and eIF4E on the functions of THP-resistant HepG2 cells was explored. After THP-treated HepG2 cells were treated with miR-15a-5p mimic and pc-eIF4E, the transfection efficacy was determined by qRT-PCR and western blot assays (Figure 4(a)), uncovering that upregulation of eIF4E counteracted the incremental level of miR-15a-5p and reduced the level of eIF4E induced by miR-15a-5p mimic. Next, the function of miR-15a-5p dependent on eIF4E was explored. The result of CCK-8 assay illustrated that miR-15a-5p mimic caused a prominent promotion in cell proliferation of HepG2 cells treated with THP, but eIF4E upregulation obviously eliminated such promotion (Figure 4(b)). EdU assay also unveiled that miR-15a-5p mimic accelerated cell growth of HepG2 cells treated with THP, and the increase could be eased when eIF4E was upregulated as evidenced by alterations in the proportion of EdU-positive cells (Figure 4(b)). Correspondingly, the inhibitory impact of miR-15a-5p mimic on THP-treated HepG2 cell apoptosis was ameliorated by eIF4E promotion (Figure 4(c)). Moreover, miR-15a-5p mimic suppressed the caspase-3 protein expression of HepG2 cells treated with THP, which was significantly reversed by eIF4E promotion (Figure 4(d)). These findings supported that downregulation of miR-15a-5p could promote the sensitivity of HepG2 cells to THP through targeting eIF4E.

## 4. Discussion

Primary hepatocellular carcinoma is one of the most common malignant tumors in China, and its mortality rate ranks the second in China [25]. Although surgical resection is the first choice for the treatment of hepatocellular carcinoma at present, it has poor postoperative effect and high recurrence rate, and most hepatocellular carcinoma has been found in the late stage and cannot be operated on [26]. Therefore, chemotherapy plays an important role in preventing the recurrence and metastasis of hepatocellular carcinoma, treating advanced hepatocellular carcinoma patients, prolonging the survival time, and improving the quality of life [27–29].

THP is a derivative of doxorubicin and is an anthracycline antitumor antibiotic synthesized from adriamycin and dihydropyran [30]. As a DNA embedment agent, THP has been shown to reduce tumor activity in hepatocellular carcinoma patients [13]. Moreover, THP has also been found to possess good inhibitory effects on many kinds of tumors, such as breast cancer and cervical cancer [14, 31]. In spite of these, the clinical application of THP is limited due to chemosensitivity resistance, which is the main cause of death in cancer patients [32]. Epidemiological survey shows that more than 90% of cancer patients die of drug resistance every year [33]. Therefore, in-depth study of the molecular mechanisms of drug resistance can provide theoretical basis for clarifying the mechanisms of drug resistance of hepatocellular carcinoma and finding new therapeutic targets.

Drug resistance of tumors is a complex process related to many factors. The abnormal expression of multiple drug resistance-related genes and the coordination of these genes lead to the appearance of drug resistance phenotype [34]. It has been found that miRNAs are involved in this process [35]. In the study, we found that miR-15a-5p was upregulated in HepG2 cells treated with THP. Studies have demonstrated that miR-15a-5p was high-expressed in resist cell lines, including NSCLC, colorectal cancer, breast cancer, and cervical carcinoma [24, 36, 37], which was in consistent with our results, suggesting that miR-15a-5p might play an essential role in the chemosensitivity resistance of hepatocellular carcinoma. To further study the effects of miR-15a-5p on the biological functions of hepatocellular carcinoma cells treated with THP, CCK-8, EdU, flow cytometry, and western blot assays were carried out. As expected, downregulation of miR-15a-5p could enhance the inhibitory effects of THP on viability and proliferation of HepG2 cells and increase the promoting effects of THP on apoptosis of HepG2 cells. There was moderate evidence suggesting positive effects of miR-15a-5p on the chemosensitivity resistance of other tumors. For example, miR-15a-5p enhances the anticancer effects of cisplatin in the resistant NSCLC cells [23]. miR-15a-5p may reverse the drug resistance in human colon cancer cells via regulating the expression of Bcl-2 [38]. Moreover, miR-15a-5p stimulates the pathogenesis and induces cisplatin chemotherapy resistance in nasopharyngeal carcinoma through targeting cyclin-dependent kinase 4 (CDK4) [39]. These findings are basically consistent with those in this study, suggesting that the downregulation of miR-15a-5p may play an important role in chemosensitivity resistance of hepatocellular carcinoma.

This study predicted that the 3′-UTR region of eukaryotic translation initiation factor 4E (eIF4E) contained complementary sites to miR-15a-5p, suggesting that eIF4E might be a target gene of miR-15a-5p. eIF4E is a key factor in the formation of protein translation initiation complex [40]. eIF4E is abnormally expressed in various cancers, including lung cancer, esophageal squamous cell carcinoma, nasopharyngeal carcinoma, gastric cancer, uterine fibroids, and breast cancer, involved in the cell growth, proliferation, invasion, and apoptosis, and closely associated with poor survival [41–43]. Furthermore, it has been found that eIF4E exhibits essential effects on chemosensitivity resistance of various cancers. For example, upregulation of eIF4E can overcome most of the resistance mechanisms arising in BRAF- (V600-) mutant cancers [44]. Hyperactive eIF4E can reduce the dependence of KRAS-mutated lung cancer cells on pemetrexed and trimetazidine [45]. eIF4E activation is critically involved in ovarian cancer chemoresistance, and inhibiting eIF4E broadly sensitizes ovarian cancer response to chemotherapy [46]. In this study, eIF4E was a target of miR-15a-5p confirmed by luciferase reporter assay and negatively associated with the expression of miR-15a-5p. Moreover, the mechanisms of miR-15a-5p/eIF4E in regulating chemosensitivity resistance of hepatocellular carcinoma cells treated with THP were further explored through restoring experiment. As expected, overexpression of eIF4E could partly restore the effects of miR-15a-5p mimic on viability, proliferation, and apoptosis of THP-treated HepG2 cells. Limitation was still needed to be addressed. Although the existing research concerning live cancer has elucidated the key regulatory role of miR-15a-5p in THP-resistant HepG2 cells, the underlying regulatory function of it *in vivo* still needs exploration. Besides, the diverse cell lines (L-02, Hep3B, and SNU-182) could be used for the following studies to in-depth validate our conclusion, since our laboratory only has the limited cell line HepG2. More studies should be conducted to make clear the function of miR-15a-5p on HCC tumorigenesis and development.

## 5. Conclusions

Our findings revealed that miR-15a-5p was upregulated in THP-resistant HepG2 cells and correlated with chemotherapy resistance via targeting eIF4E, providing an experimental basis that miR-15a-5p might act as a novel diagnostic target in hepatocellular carcinoma resistance to THP.

## Figures and Tables

**Figure 1:** miR-15a-5p is upregulated in THP-treated HepG2 cells. The expression of miR-15a-5p in HepG2 cells treated with THP was detected by qRT-PCR assay. ^∗∗^*P* < 0.01 vs. the HepG2 group. All data were presented as mean ± SD. *n* = 3.

**Figure 2:** Downregulation of miR-15a-5p blocks cell growth and elevates cell apoptosis in THP-treated HepG2 cells. (a) qRT-PCR assay was performed to evaluate the miR-15a-5p expression in THP-treated HepG2 cells after transfection with miR-15a-5p inhibitor. (b) The viability and proliferation of THP-treated HepG2 cells transfected with miR-15a-5p inhibitor were assessed by CCK-8 and EdU assays. (c) The apoptosis of THP-treated HepG2 cells transfected with miR-15a-5p inhibitor was evaluated by flow cytometer. (d) The caspase-3 protein level in THP-treated HepG2 cells transfected with miR-15a-5p inhibitor was evaluated by western blot assay. ^∗∗^*P* < 0.01 vs. the HepG2 group; ^#^*P* < 0.05 and ^##^*P* < 0.01 vs. HepG2+THP+inhibitor of the NC group. All data were presented as mean ± SD. *n* = 3.

**Figure 3:** eIF4E is a target gene of miR-15a-5p and negatively associated with miR-15a-5p expression. (a) The target gene of miR-15a-5p was predicted with ENCORI and miRwalk. ^∗∗^*P* < 0.01 vs. the NC inhibitor group. (b) Binding sites between miR-15a-5p and eIF4E. (c) Luciferase reporter analysis was employed to validate the interactions between miR-15a-5p and eIF4E. ^∗∗^*P* < 0.01 vs. the NC mimic group. (d) qRT-PCR and (e) western blot assays were performed to evaluate the eIF4E expression in HepG2 cells after transfection with miR-15a-5p inhibitor. ^∗∗^*P* < 0.01 vs. the NC inhibitor group. All data were presented as mean ± SD. *n* = 3.

**Figure 4:** eIF4E mediates the effects of miR-15a-5p on the THP chemoresistance of HepG2 cells. (a) qRT-PCR and western blot assays were performed to evaluate the miR-15a-5p and eIF4E protein expressions in THP-treated HepG2 cells transfected with miR-15a-5p mimic or pc-eIF4E. (b) The viability and proliferation of THP-treated HepG2 cells transfected with miR-15a-5p mimic or pc-eIF4E were assessed by CCK-8 and EdU assays. (c) The apoptosis of THP-treated HepG2 cells transfected with miR-15a-5p mimic or pc-eIF4E was evaluated by flow cytometer. (d) The caspase-3 protein level in THP-treated HepG2 cells transfected with miR-15a-5p mimic or pc-eIF4E was evaluated by western blot assay. ^∗^*P* < 0.05 and ^∗∗^*P* < 0.01 vs. the HepG2 group; ^#^*P* < 0.05 and ^##^*P* < 0.01 vs. the HepG2+THP+miR-NC+pc-NC group; ^&&^*P* < 0.01 vs. the HepG2+THP+miR-15a-5p mimic+pc-NC group. All data were presented as mean ± SD. *n* = 3.

## Data Availability

The data used during the present study are available from the corresponding author upon reasonable request.
